# Ship Target Detection in Optical Remote Sensing Images Based on Multiscale Feature Enhancement

**DOI:** 10.1155/2022/2605140

**Published:** 2022-10-06

**Authors:** Liming Zhou, Yahui Li, Xiaohan Rao, Cheng Liu, Xianyu Zuo, Yang Liu

**Affiliations:** ^1^Henan Key Laboratory of Big Data Analysis and Processing, Henan University, Kaifeng, Henan, China; ^2^School of Computer and Information Engineering, Henan University, Kaifeng, Henan, China; ^3^Henan Province Engineering Research Center of Spatial Information Processing and Shenzhen Research Institute, Henan University, Kaifeng 475004, China

## Abstract

Due to the multiscale characteristics of ship targets in ORSIs (optical remote sensing images), ship target detection in ORSIs based on depth learning is still facing great challenges. Aiming at the low accuracy of multiscale ship target detection in ORSIs, this paper proposes a ship target detection algorithm based on multiscale feature enhancement based on YOLO v4. Firstly, an improved mixed convolution is introduced into the IRes (inverted residual block) to form an MIRes (mixed inverted residual block). The MIRes are used to replace the Res (residual block) in the deep CSP module of the backbone network to enhance the multiscale feature extraction capability of the backbone network. Secondly, for different scale feature maps' perception fields, feature information, and the scale of the detected objects, the multiscale feature enhancement modules—SFEM (small scale feature enhancement module) and MFEM (middle scale feature enhancement module)—are proposed to enhance the feature information of the middle- and low-level feature maps, respectively, and then the enhanced feature maps are sent to the detection head for detection. Finally, experiments were implemented on the LEVIR-ship dataset and the NWPU VHR-10 dataset. The accuracy of the proposed algorithm in ship target detection reached 79.55% and 90.70%, respectively, which is improved by 3.25% and 3.56% compared with YOLO v4.

## 1. Introduction

Target detection is important in military and civilian fields and has a wide range of application scenarios. Traditional target detection algorithms are mostly based on sliding windows and artificial feature extraction. Although it has achieved good results, there are still a series of deficiencies. Firstly, the method based on sliding window has high running cost and time complexity. Secondly, the robustness of manually designed features is poor [1–3]. Upon the development of deep learning, target detection methods based on deep learning have gradually replaced traditional methods. Many representative natural image target detection algorithms have been proposed and widely used, such as R-CNN [4], fast R-CNN [5], faster R-CNN [6], SSD [7], and YOLO [8–10] series.

As an important technology of ocean monitoring, ship target detection is significant in national security and maritime transportation safety. With the development of aerospace technology, ORSIs data are increasing. Therefore, more and more scholars try to apply the natural image target detection algorithm to ship detection in ORSIs. However, unlike natural images, ship detection in ORSIs is more difficult. As shown in Figure 1, the large field of view and the small ship target in Figure 1(a) cause a huge difference in the ratio of foreground pixels and background pixels of the ship target, which increases the difficulty of detection. In Figure 1(b), the texture and clarity of the shadow-affected ships are poor in the case of cloud and shadow occlusion. The small, medium, and large ships in Figure 1(c) have poor contrast between the foreground and background due to the influence of the wave background and wake [11]. Therefore, ship target detection in ORSIs still faces great challenges.

In ORSIs, large field of view, low resolution, and complex background make the detection precision of large, medium, and small ships generally low. Therefore, how to improve the detection precision of multiscale ship targets has become a research hotspot of scholars. Zhou et al. [12] proposed the MSSDNet (multiscale ship detection network). Firstly, CSPMRes2 (cross stage partial network with modified Res2Net) is used as the basic module of the backbone network for multiscale feature extraction. Secondly, FC-FPN (feature pyramid network with fusion coefficients) is used for multiscale feature adaptive fusion. The multiscale ship detection accuracy of this method has reached an advanced level. However, compared with the baseline network, the network introduces a large number of parameters and computation, the reasoning speed is only half of the baseline network, and the model size is about 1.7 times of the baseline network. Zhou et al. [13] proposed a ship object detection method based on feature enhancement. It uses the EIRM (elastic inception residual module) module to perform feature enhancement on the low- and middle-level feature maps. EIRM module extracts the feature information of multiscale ship targets through scaling strategy and uses SGPANet for further extraction and fusion of multiscale features. This method only adds a small amount of parameters relative to the baseline network. Wang et al. [14] proposed the FSoD-Net (full-scale object detection network). Firstly, a wider backbone network is proposed for feature extraction. For different scale feature maps, it adopts different feature extraction modules and regression layers. This method has achieved advanced performance in full-scale target detection in ORSIs.

According to the above analysis, aiming at the problem that it is difficult to detect multiscale ship targets in ORSIs, this paper proposes a ship target detection method based on multiscale feature enhancement based on YOLO v4 [15]. Experiments on the LEVIR-ship and NWPU VHR-10 datasets show that the proposed method achieves better results than YOLO v4. The main contributions of this paper are summarized as follows:

1. The MIRes are proposed and applied to the deep layers of the backbone network. Firstly, to enhance the feature extraction ability of the backbone network, the Res in the deep CSP module of the backbone network is replaced by the IRes. Secondly, to extract the multiscale feature information of the ship target, the mixed convolution is improved and the depthwise separable convolution of the IRes is replaced by the modified mixed convolution.
2. Two multiscale feature enhancement modules, SFEM and MFEM, are proposed for different size feature maps to enhance the features of low- and middle-level feature maps, respectively. SFEM and MFEM act on feature maps of 52 × 52 and 26 × 26 scales, respectively, and use atrous convolutions with different dilation rates to enhance the receptive field of feature maps while extracting information.
3. Experiments on the LEVIR-ship dataset show that the proposed method achieves higher accuracy in the detection of multiscale ships in ORSIs. Simultaneous ablation experiments demonstrate the benefit of all partial improvements in this paper. The extended experiments on the NWPU VHR-10 dataset show that the method in this paper can achieve good results on different datasets and different categories.

This paper is organized as follows: Section 2 reviews some related work.  Section 3 introduces the proposed method in detail.  Section 4 is the experimental part, including comparative experiments and ablation experiments.  Section 5 gives the conclusion.

## 2. Related Work

### 2.1. One-Stage Detection Algorithm Backbone Network

With the development of convolutional neural network classification techniques, scholars have proposed deeper networks for classification tasks, such as ResNet50 [16], Darknet53 [10], and ResNet-101 [16]. These deep networks have powerful feature extraction capabilities, so they are widely used in the backbone network of target detection. Although the deep convolutional neural network has strong robustness, a large number of convolutions will cause the loss of small target pixels and the destruction of texture structure, so its applicability for small target detection is poor.

Qi et al. [17] used the YOLO v3 framework with auxiliary networks for object detection. The auxiliary network is lighter than the backbone network and has fewer convolutions, so it can retain more location information. The backbone network and auxiliary network extract features at the same time, and the location information extracted from the auxiliary network is transmitted to the backbone network. The combination of the deep semantic information extracted by the backbone network and the location information extracted by the auxiliary network greatly improves the detection accuracy of the network. Qing et al. [18] used the improved RepVgg as the backbone network for feature extraction. The backbone network uses multibranch structure for feature extraction during training, and each convolution is followed by a residual connection to accelerate the convergence of the network. At the same time, considering multiple branches will increase inference time, so only single-branch structure is used when inference. Then, the neck network uses the improved FPN [19] for feature fusion and finally uses four scales for detection, which achieves good detection results. Xu et al. [20] used a densely connected network (DenseNet) to enhance the feature extraction ability of YOLO v3 backbone network for poor detection accuracy in ORSIs object detection. Then, some of the residual blocks in the third and fourth residual units of the Darknet53 backbone network are replaced by dense connection blocks. Finally, four detection heads are used for detection, and the detection accuracy is significantly improved.

Sandler et al. [21] explored the impact of bottleneck structure on accuracy and parameters, proposed IRes (inverted residual block), and built a lightweight MobileNet V2 network based on the IRes. The structure of the IRes makes the feature extraction part have a wider channel and can extract richer feature information. Meanwhile, the introduction of depthwise separable convolution makes the module lightweight. Although depthwise separable convolutions tend to cause the problem of accuracy degradation, the wider structure makes up for this shortcoming. Tan et al. [22] discussed the effect of different convolution kernel sizes on network performance, proposed mixed convolution, and built MixNet using mixed convolution for natural image target detection. Different from traditional convolution, mixed convolution divides the input channels into different groups, then each group corresponds to a depthwise separable convolution with different kernel sizes, and finally fuses the outputs of each convolution. Mixed convolution introduces different convolution operations in a single convolution, so it can extract feature information of different scales from a single feature map while reducing part of the amount of computation and parameters.

### 2.2. Feature Enhancement Module

To solve the problem that multiscale targets are difficult to detect ORSIs, researchers have applied feature pyramids such as FPN [19] and PANet [23] for multiscale detection. Zhang et al. [24] found that there was a problem with the simple fusion of feature pyramids, so they proposed a multilevel feature pyramid. Firstly, they used CAFUS (content-aware feature upsampling) instead of upsampling to solve the fusion problem of feature maps of different scales. Then, FEM (feature enhancement module) is proposed to enhance the fused feature map. Wang et al. [25] proposed SE-SSD (spatial enhanced single shot multi box detector). Firstly, the spatial information is enhanced by increasing the number of image channels. Secondly, the output of the backbone network is modified, and a pooling operation is removed. Finally, a context feature enhancement module is designed to act on the middle and low layer feature maps to enhance the receptive field of the middle and low layer feature maps. Wang et al. [26] proposed an improved YOLO v3 algorithm for multiscale object detection. Dense connection blocks are used instead of residual units in Darknet53 to enhance the feature extraction capability of the backbone network. The feature enhancement module is proposed to act on the middle- and low-level feature maps to enhance the location information contained in the shallow feature maps. Finally, the FPN is improved. This method significantly improves the detection accuracy of small targets in ORSIs.

Liu et al. [27] proposed a lightweight RFB inspired by the human receptive field. RFB mainly includes two parts: multibranch structure and atrous convolution [28]. Each branch structure contains convolution kernels of different sizes and atrous convolutions with different expansion rates. The original RFB structure mainly consists of three branches, each of which contains a convolution kernel of 1 × 1, 3 × 3, and 5 × 5, corresponding to dilated convolutions with expansion rates of 1, 3, and 5, respectively. The convolution kernels of different sizes can better simulate the receptive field and extract feature information, which is significantly better than the convolution kernel of fixed size. Atrous convolution can capture feature information in larger regions without increasing parameters.

Although the above methods have achieved good detection accuracy, Chen et al. [29] pointed out that the key to the feature fusion pyramid is to divide and conquer, so it only uses a single-layer feature map for detection. However, single-layer feature maps have poor detection accuracy for small objects. Therefore, this paper retains PANet for multiscale feature map fusion and then uses different modules for feature enhancement of different scale feature maps to improve the accuracy of multiscale ship detection.

## 3. Methodology

In this section, the algorithm proposed in this paper is introduced in detail through four sections: Section 3.1;overall network structure; Section 3.2;backbone with MIRes; Section 3.3;PANet with multiscale feature enhancement; and Section 3.4;LOSS function.

### 3.1. Overall Network Structure

The overall network structure of the algorithm in this paper is shown in Figure 2. The network mainly consists of four parts: the CSP Darknet53 backbone network is used for feature extraction, the PANet neck network is used for feature fusion, MSFE is used for multiscale feature enhancement, and the YOLO Head is used for detection. The backbone network contains five CSP modules (C1–C5). C1–C4 contain different numbers of residual blocks (1,2,8,8), and C5 contains four MIRes. Among them, the 13 × 13 and 26 × 26 feature maps extracted by the third and fourth CSP modules are directly used as the input of PANet. The feature map of size 52 × 52 extracted by the fifth CSP module first passes through the SPP module and then is input into PANet for feature fusion. PANet fuses feature maps of different scales through upsampling and downsampling. After the feature maps are fused by PANet, the 13 × 13 and 26 × 26 scale feature maps are sent to the detection head together with the 52 × 52 scale feature maps through the multiscale feature enhancement modules—SFEM and MFEM—for detection. Algorithm 1 describes the basis idea of multiscale feature enhanced ship target detection.

Figure 3 is the structure of the SPP module. In the SPP module, the input feature map first goes through three different sizes of max pooling layers (5, 9, 13), and then the output of each pooling layer is fused with the input feature map. The SPP module was proposed for input image resizing [30]. In this paper, it is mainly used to increase the reception range of backbone features and separate context features.

Figure 4 shows the CSP module structure. In the CSP structure, the input feature map is sent to two branches of different depths, and the branch containing Res × *N* is responsible for feature extraction, and then directly fused with another branch. The CSP module can improve the accuracy of the model while reducing weight.

### 3.2. Backbone with MIRes

The amount of feature information is closely related to the accuracy of object detection, and the C5 feature map of the CSP Darknet53 backbone network contains generous contextual feature information [31]. Therefore, this paper considers to enrich the feature information of C5 by improving the feature extraction capability of the fifth CSP module to improve the accuracy of multiscale ship target detection. At present, many researchers improve the feature extraction ability of the network by increasing the depth, but the increase of the depth is always accompanied by a surge in the amount of computation. Therefore, in order not to increase the redundant computation, this paper considers increasing the width of the network instead of the depth.

The wider network structure of the IRes enables it to have strong feature extraction capabilities, and the presence of depthwise separable convolutions makes it lightweight enough. However, for multiscale ship detection, it still lacks the ability to extract multiscale features. Therefore, this paper proposes MIRes, which introduces an improved mixed convolution into the IRes. The MIRes are used to replace the Res in the fifth CSP module, which greatly improves the multiscale feature extraction capability of the backbone network with a small increase in the amounts of parameters and computation.

The MIRes structure is shown in Figure 5, where MC is a mixed convolution and *c* is the channels number. MIRes adopts the IRes structure, and the number of network channels is expanded by 6 times compared with Res. Channel extended mixed convolution is used for multiscale feature extraction.  Table 1 shows the network architecture and parameters of Res and MIRes.

For the same input, we can use a simple formula to show the difference in the output feature maps of mixed convolution and depthwise separable convolution. In this case, the input feature map size h (height) and *w* (width) are equivalent and the output feature map size is the same. Assuming that a depthwise separable convolution isW^(k, k, c, m)^, Y^(h, w, c∙m)^ is the output tensor. Then, each output feature map can be represented by the following formula (1). Different from the depthwise separable convolution, if the mixed convolution input channels are divided into *g* groups, the number of input and output channels is equal. Similarly, the convolution kernels are also divided into *g* groups. Then, the output for the t-th group can be expressed in formula (2). The total output of the mixed convolution can be represented in formula (3).1

(1) $$\begin{array}{c} Y_{x,y,z}=\underset{-\frac{k}{2}\leq i\leq \frac{k}{2},-\frac{k}{2}\leq j\leq \frac{k}{2}}{\sum }X_{x+i,y+j,z/m}∙W_{i,j,z}\forall_{z}=1,\cdots ,m∙c\text{,} \end{array}$$

(2) $$\begin{array}{c} {\hat{Y}}_{x,y,z}^{t}=\underset{-\frac{k_{t}}{2}\leq i\leq \frac{k_{t}}{2},-\frac{k_{t}}{2}\leq j\leq \frac{k_{t}}{2}}{\sum }{\hat{X}}_{x+i,y+j,z/m}^{t}∙{\hat{W}}_{i,j,z}^{t}\forall_{z}=1,\cdots ,m∙c_{t}\text{,} \end{array}$$

(3) $$\begin{array}{c} Y_{x,y,z_{0}}=\text{Concat}\left({\hat{Y}}_{x,y,z_{1}}^{1},\cdots {\hat{Y}}_{x,y,z_{g}}^{g}\right)\text{.} \end{array}$$

In formula (1), *k* × *k* is the size of the convolution kernel, c is the input channel, and m is the channel multiplier. In formula (2) $\langle {\hat{X}}^{\left(h,w,c_{1}\right)},\cdots {\hat{X}}^{\left(h,w,c_{g}\right)}\rangle$ is the mixed convolution channel of group *g*, and $\langle {\hat{W}}^{\left(k_{1},k_{1},c_{1},m\right)},\cdots {\hat{W}}^{\left(k_{g},k_{g},c_{g},m\right)}\rangle$ is the depthwise separable convolution channel of group *g*. In formula (3), z_0_=z_1_, +⋯+z_g_=m∙c。

ORSIs have a large field of view, and most ship targets have small foreground pixels. Large kernel convolution can easily cause the loss of target pixels and bring a lot of computation. Therefore, we have improved the kernel size of the mixed convolution and changed the way the number of channels is divided.  Figure 6 shows the proposed mixed convolution structure. Firstly, we removed the 9 × 9 convolution to avoid the problem of information loss during the convolution process. Secondly, a 1 × 1 convolution is added, which further reduces the amount of computation and parameters on the basis of retaining more detailed feature information. Finally, we abandon the equal distribution and choose the exponential distribution for channel partitioning of convolutions with different kernel sizes. The latter retains more low-latitude feature information while realizing multiscale feature extraction. Compared with the method of using equal division between channels in natural images, the performance of exponential division in ORSIs is higher. The exponential channel division method is shown as follows:

(4) $$\begin{array}{c} C_{x}=\left\{\begin{array}{c} 2^{-x},0<x<i-1\text{,}\\ 2^{-x+1},x=i\text{,} \end{array}\right. \end{array}$$

where i is the number of convolution kernels and C_x_ is the number of channels of the x-th convolution. According to the parameters in Table 1 and formula (3), the output feature map of the proposed mixed convolution can be expressed by the following formula:

(5) $$\begin{array}{c} Y_{13,13,3072}=\text{Concat}\left({\hat{Y}}_{1,1,1536}^{1},{\hat{Y}}_{3,3,768}^{2},{\hat{Y}}_{5,5,384}^{3},{\hat{Y}}_{7,7,384}^{4}\right)\text{.} \end{array}$$

MIRes has a wider network structure and introduces mixed convolution, so the multiscale feature extraction capability of the network is greatly improved At the expense of a small amounts of parameters (Parameter 9M) and computation (BFLOPS 0.759 G), MIRes greatly enhance the multiscale feature extraction capability of the backbone network, and the detection accuracy of multiscale ship targets is significantly improved (2.45%).

### 3.3. PANet with Multiscale Feature Enhancement

PANet is the mainstream solution for multiscale target detection. It is based on a rule: shallow feature maps (C3) contain higher resolution and more location information, and deep feature maps (C5) have larger receptive field and more semantic information [32]. The shallow receptive field is smaller, and its location information is more beneficial to target localization. The deep receptive field is larger, which contains more semantic information, which is beneficial to the classification of objects. Take Figure 7 as an example. The shallow network (C3) contains more local information, that is, fine-grained information, and the receptive field at this time is relatively small. Therefore, the local information of the feature map obtained by the shallow network is relatively rich, the resolution of the feature map at this level is relatively high, and the receptive field of a single pixel is relatively small, which can capture more location information. As the number of downsampling or convolution increases, the deep feature (C5) gradually increases the receptive field and the overlapping area between the receptive fields. The information represented by the pixels at this time is the information of a region, and the feature information obtained is the feature information between this region or adjacent regions, which is relatively not fine-grained and low in resolution, but rich in semantic information [33, 34]. The feature information extracted by MIRes first passes through the SPP module and then is input into PANet for fusion. In PANet, the deep feature map is fused with the upper layer feature map in a ratio of 1 to 1 after upsampling, so that the deep semantic information is transferred to the shallow feature map. The feature map of the shallow layer is fused with the feature map of the next layer in a ratio of 1 after downsampling, so that the position information of the shallow layer is transmitted to the deep layer. This fusion mode can improve the accuracy of multiscale target detection, but for small- and medium-sized ship targets, this simple fusion strategy may not be able to adapt to the multiscale characteristics of ship targets in remote sensing images. Therefore, this paper further improves the accuracy of multiscale ship target detection by enhancing the feature information of the middle- and low-level feature maps.

The receptive field mechanism of RFB can significantly enhance the receptive field and feature information of feature maps. However, there are still problems when RFB is directly applied to ship target detection in ORSIs. The large convolution cores and large expansion rates in RFBs may cause target miss and misdetection for small- and medium-sized ships. Therefore, for the appeal problems, this paper proposes multiscale feature enhancement modules: SFEM and MFEM. For low-level feature maps, SFEM introduces a multibranch structure and uses ordinary convolution and atrous convolution with an expansion rate of 1 for feature extraction. For the midlevel feature maps, feature enhancement is performed using MFEM containing atrous convolutions with large expansion rates. Considering the parameters of the network at the same time, different from other deep feature enhancement modules, we abandon the deeper network structure and use a wider network for multiscale feature extraction. Finally, considering that the input and output of the SFEM and MFEM modules do not involve channel transformation, the 1 × 1 convolution used to adjust the dimension.

For the low-level feature map, it is mainly responsible for the detection of small-scale ship targets. For small targets, too large receptive field will introduce a large amount of background, resulting in the decline of detection accuracy. Therefore, in this paper, the atrous convolution with a large expansion rate is replaced by an ordinary 3 × 3 convolution, and only ordinary convolution and atrous convolution with an expansion rate of 1 are used to extract features. At the same time, the 5 × 5 large kernel convolution branch is removed and a 3 × 3 convolution branch is added.  Figure 8 shows the structure of SFEM. *R* represents the dilation rate of the atrous convolution, and shortcut represents the residual connection. The input feature map goes through four-branch structure for feature extraction. Each branch contains the same input, and the feature information extracted by each branch is fused and added to the input feature map. Compared with the RFB module, SFEM can enhance the shallow position information while reducing the introduction of noise, effectively improving the accuracy of ship detection.

For the midlevel feature map, it needs appropriate receptive field for the detection of medium-scale ship targets. Therefore, we use a combination of standard convolution and atrous convolution to extract features. Its structure is similar to SFEM. On the basis of retaining the multibranch structure, atrous convolution is used to enhance the receptive field and capture a wider range of feature information.  Figure 9 shows the structure of MFEM. *R* is the dilation rate of atrous convolution, and shortcut is the residual connection. MFEM retains the network structure of SFEM and the atrous convolution with large expansion rate in RFB, which can enhance the receptive field of the effective area while maintaining the size of the feature map.

SFEM and MFEM can enhance the feature description of multiscale ship targets and improve the accuracy of ship detection. At the same time, it can achieve better results than some more advanced enhancement modules such as RFB and EIRM [13]. In Section 4, a series of comparative experiments are implemented to verify the effectiveness of the module.

### 3.4. Loss Function

The feature map after feature enhancement is predicted at the detection head. The three prediction scales of the algorithm in this paper are 13 × 13, 26 × 26, *an* *d* 52 × 52. During prediction, the feature map is divided into *S* × *S* grids, and each grid will contain multiple prediction boxes. The final result is obtained by calculating the joint intersection of IOU [35] and then filtering with nonmaximum suppression (NMS). In this paper, the CIOU [36] loss function is used to calculate the bounding box regression loss, and the loss functions such as GIOU [37], DIOU, and IOU are compared.

The IOU loss function is usually used to calculate the bounding box regression loss, the intersection-over-union (IOU). Assuming that the predicted box is defined asB_pre_ and the ground-truth box is defined asB_gt_, the IoU loss function (7) is as follows:

(6) $$\begin{array}{c} IOU=\frac{\left|B_{pre}\cap B_{gt}\right|}{\left|B_{pre}\cup B_{gt}\right|}\text{,} \end{array}$$

(7) $$\begin{array}{c} L_{IOU}=1-\frac{\left|B_{pre}\cap B_{gt}\right|}{\left|B_{pre}\cup B_{gt}\right|}\text{.} \end{array}$$

However, as shown in Figure 10, there are still problems with the IOU loss function. Firstly, when B_pre_ and B_gt_do not intersect, IOU=0. Secondly, when the twoB_pre_ are not the same, the two IOUs are equal.

To solve the problem of IOU=0 when the predicted frame and the real frame do not intersect, GIOU introduces the minimum bounding box based on the predicted frame and the real frame. Assuming that the predicted frame is B_pre_, the real frame isB_gt_, and A_c_ is the minimum bounding box, GIOU can be expressed by

(8) $$\begin{array}{c} G_{IOU}=IOU-\frac{\left|A_{c}-B_{pre}\cap B_{gt}\right|}{\left|A_{c}\right|}\text{.} \end{array}$$

However, when the predicted box and the ground-truth box input contain relationship, GIOU will degenerate into IOU, which still has the problem of equal IOU. DIOU is based on IOU and GIOU, taking into account the distance between the ground-truth box and the predicted box, and can guide the direction movement of the prediction box when the two do not intersect. The DIOU loss function formula is as follows:

(9) $$\begin{array}{c} DIOU=IOU-\frac{\rho^{2}\left(b,b_{gt}\right)}{c^{2}}\text{.} \end{array}$$

In formula (9), *b* and b_gt_ are the center points of the prediction madness and the real box, respectively,*ρ*represents the Euclidean distance between the two center points, and *c* is the diagonal length of the minimum bounding box between the real box and the prediction box. The DIOU parameters are shown in Figure 11. According to Figure 9, it can be seen that when the target box completely includes the prediction box, GIOU will completely degenerate into IOU. Therefore, GIOU cannot converge well in advanced algorithms, thus affecting the detection accuracy. And, DIOU adds a penalty term*ρ*^2^(*b*, *b*_*gt*_)/*c*^2^on the basis of GIOU. It can minimize the normalized distance between the center points of the two bounding boxes, while the diagonal is unchanged, so that it converges faster than GIOU.

Three important factors for bounding box regression loss are overlap area, center point distance, and aspect ratio. DIOU ignores the key factor of aspect ratio. CIOU considers the aspect ratio of the predicted box and the ground-truth box, which can be well adapted to the aspect ratio characteristics of the ship target. The CIOU formula is as follows:

(10) $$\begin{array}{c} \begin{array}{c} CIOU=\frac{\rho^{2}\left(b,b_{gt}\right)}{c^{2}}+\alpha \upsilon \text{,}\\ \alpha =\frac{\upsilon }{\left(1-IOU\right)+\upsilon }\text{,}\\ \upsilon =\frac{4}{\pi^{2}}{\left(\tan^{-1}\frac{w^{gt}}{h^{gt}}-\tan^{-1}\frac{w}{h}\right)}^{2}\text{.} \end{array} \end{array}$$

In the above formulas,*α*is a positive parameter. *υ*means consistency of aspect ratio.*w*^*gt*^ and *h*^*gt*^ are the width and height of the real box, and *w* and *h* are the width and height of the predicted box.

## 4. Experiments and Results

To verify the proposed method, a series of experimental comparisons are implemented in this section. In Sections 4.1, 4.2, and 4.3, the dataset, experimental details, and evaluation indicators are introduced. In Section 4.4, a comparative experiment is implemented to compare with other algorithms and the baseline network. Section 4.5 is the ablation experiment. Section 4.6 is an extended experiment.

### 4.1. Dataset

The LEVIR dataset contains a large number of background images (that is, images that do not contain objects), so we segment the LEVIR dataset to form the LEVIR-ship dataset. The LEVIR-ship dataset only retains images containing ship targets for ablation experiments and comparative experiments to verify the superiority of the proposed algorithm in multiscale ship target detection. The NWPU VHR-10 dataset has various categories, the target scale changes greatly, and the target distribution is relatively concentrated, which is very challenging. Therefore, we conduct extended experiments on the NWPU VHR-10 dataset to verify the applicability and scalability of the proposed algorithm for different datasets and different targets. We will give a detailed introduction to the LEVIR-ship and NWPU VHR-10 datasets, respectively.

The LEVIR [38] dataset contains a total of 21,952 images with a resolution of 600 × 800 pixels. There are three categories: aircrafts, ships, and storage tanks. We separate out the ship categories and remove images that do not contain objects to form the LEVIR-ship dataset. LEVIR-ship has a total of 1494 images and 3025 ship targets, and each image contains at least one ship target. According to the original partitioning method, the training set contains 876 images of 1790 ship targets, and the test set contains 618 images of 1235 ship targets. The target location distribution and scale distribution in the LEVIR-ship dataset are shown in Figure 12. In Figure 12(a), the horizontal axis and the vertical axis are the positions of the target in the width and height of the image, respectively, the horizontal axis in Figure 12(b) is the target pixel, and the vertical axis is the number of targets. It is obvious that the target location distribution and scale distribution in the lever ship data set are relatively uniform.

The NWPU VHR-10 [39] dataset contains a total of 800 high-resolution images and ten classes of objects. In this paper, 150 background images without targets are deleted, and 650 images with targets are reserved for training and testing. The training set and test set are randomly divided in a ratio of 5 to 5.  Figure 13 shows the target location distribution and scale distribution in the NWPU VHR-10 dataset. In Figure 13(a), the horizontal axis and the vertical axis are the positions of the target in the width and height of the images, respectively, the horizontal axis in Figure 13(b) is the target pixel, and the vertical axis is the number of targets. Most of the objects in the NWPU VHR-10 dataset are gathered in the central area of the images, and there are few small-scale objects, mostly medium-scale targets.

### 4.2. Implementation Details

Before training, the images are resized to 416 × 416 size and then sent to the network for training. The training has a total of 4000 iterations. The training batch size is set to 64, and the initial learning rate is 0.0001. When iterating to 3200 and 3600 times, the learning rate is reduced by one tenth, respectively. The training of the network was performed on an RTX3060 GPU, and the training was accelerated using CUDA 11.3 and cuDNN 8.05.

The algorithm in this paper performs location and category regression based on predefined anchor boxes on *S* × *S* grids of each image. Therefore, the generation of anchor boxes has a great impact on the performance of the network. The K-means++ algorithm can generate better anchor boxes to accelerate the convergence of the network. In order to speed up the convergence of the network, this paper uses the K-means++ clustering algorithm to obtain the size of the prior box. The clustering process of the K-means++ algorithm is shown in Algorithm 2. The size of the prior box is shown in Table 2. Each prediction scale sets three prior frames, which are, respectively, suitable for the detection of large, medium, and small objects.

### 4.3. Evaluation Criteria

In this paper, the general evaluation methods map and FPs are used to evaluate the algorithm. The mAP is a general evaluation criterion in object detection, which is determined by *P* (precision) and *R* (recall). The formulas for calculating P and *R* are as follows:

(11) $$\begin{array}{c} P=\frac{TP}{TP+FP}\text{,} \end{array}$$

(12) $$\begin{array}{c} R=\frac{TP}{TP+FN}\text{.} \end{array}$$

In formula (13) and formula (14), TP represents positive samples, that is, the number of ships detected; FP represents the negative sample, that is, the number of ships incorrectly detected; FN stands for false samples, that is, the number of ships missed [40]. According to *P* and *R,* the calculation of mAP can be expressed as follows:

(13) $$\begin{array}{c} mAP=\frac{\sum_{i=1}^{N_{cls}}\int P_{i}\left(R_{i}\right)dR_{i}}{N_{cls}}\text{.} \end{array}$$

In the above formula, N_cls_ represents the number of categories in the dataset.P_i_ represents the precision of the i-th class, and R_i_ represents the recall of the i-th class. In this paper, FPS is used to evaluate the inference speed of the algorithm. The FPS formula is

(14) $$\begin{array}{c} FPS=\text{frameNumelapsedTime.} \end{array}$$

In the above formula, frameNum is the number of images, and elapsedTime is the inference time. The higher FPS indicates that the model inferences faster.

### 4.4. Comparative Experiments

In this section, the comparison experiment is divided into two parts. In Section 4.4.1, the proposed algorithm is compared with other methods and baseline network, and the advantages of this algorithm are analyzed. In Section 4.4.2, the feasibility of this improvement is compared. The improvement feasibility comparison mainly includes the feasibility of mixed convolution improvement, the comparison of Res, and the comparison of feature enhancement modules (SFEM and MFEM) with RFB and EIRM.

#### 4.4.1. Comparison with Other Methods and Baseline Network

According to the experimental parameter settings in Section 4.2, a comparative experiment was conducted on the lever ship data set, and the results are shown in Table 3. First, compared with the baseline network, the improvement of the algorithm in this paper has achieved better results. Although the detection speed (FPS) decreased slightly, the accuracy of multiscale ship detection was improved by 3.25%. Secondly, compared with other two-stage algorithms, the mAP and FPS of this algorithm have reached the highest level. In general, the accuracy of the proposed algorithm has been greatly improved compared with the baseline network, and the speed still has great advantages compared with the two-stage algorithm, meeting the requirements of real-time detection (*FPS* ≥ 30).

Figure 14 is a comparison chart of the loss function curve between YOLO v4 and the algorithm in this paper. The blue is the loss value curve, and the red is the mAP curve. The loss curve represents the difference between the predicted and actual results. According to the loss curve and mAP curve, it is obvious that the proposed algorithm converges faster than YOLO v4, and the loss value is lower and the accuracy is higher. The model in this paper is significantly better than the YOLO v4 network in terms of detection accuracy.

Figure 15 is a comparison chart of the detection results between the algorithm in this paper and the YOLO v4 algorithm. In order to make the detection results more representative, we selected a total of six groups of images for comparison. Among them, Figures 15 (a)–15 (g) is the original image, Figures 15 (h)–15 (n) is the detection result of YOLO v4, and Figures 15 (o)–15 (u) is the detection result of the proposed algorithm. In Figure 14, the images Figures 15 (a)–15 (c) contain small, medium, and large-scale ship targets; in Figure , the ship targets have long wakes and complex wave backgrounds; in Figure 15 (f), the ship targets are occluded by shadows; in Figure 15 (g), the ship target is affected by strong light and the contrast between light and dark is strong. According to the characteristics of the above images and the detection results of Figures 15 (h)–15 (n), it can be seen that the feature extraction ability and the receptive field of the feature map of YOLO v4 algorithm are obviously insufficient, which is easy to cause missed detection and false detection of multiscale ships. According to Figures 15 (o)–15 (u), it is obvious that the proposed algorithm has high detection accuracy in multiscale ship detection and can detect large, medium and small-scale ship targets well. At the same time, under the influence of wake, wave background, light, and shadow, the algorithm in this paper can well suppress the interference of background factors and accurately detect ship targets of various scales.

#### 4.4.2. Comparison of the Baseline Network and the Proposed Method

In order to verify the influence of the size of the convolution kernel and the channel allocation method on the detection accuracy, in this paper, different convolution kernels and assignment methods are used to perform ablation experiments. The experimental results are shown in Table 4. 1357exp means that the convolution kernels are 1, 3, 5, and 7, and the channels are divided in the exponential form. 1357 means that the convolution kernels are 1, 3, 5, and 7, and the channels are divided equally. At the same time, we added two evaluation indicators—Parameter and BFLOPS. Parameter represents the size of the model, that is, the amount of parameters, and BFLOPS represents the amount of model calculation. According to the results, it can be seen that removing the large kernel convolution and replacing it with a 1 × 1 convolution can bring a little improvement in accuracy, while the amounts of parameters and calculation are also slightly reduced. In the comparison between the exponential division and the equal division, the exponential division achieves higher accuracy. Therefore, for the multiscale ship detection of ORSIs, due to the complexity of ORSIs and the multiscale characteristics of ship targets, compared with large kernel convolution, 1 × 1 convolution may be more efficient. The comparison results verify that the improvement of the mixed convolution in this paper enables it to achieve excellent results in multiscale ship detection in ORSIs.

To verify the superiority of the proposed MIRes, the influence of various residual blocks on the detection accuracy is compared in this paper.  Table 5 shows the comparison results of various residual blocks. It is obvious that although IRes has better feature extraction ability, its accuracy has been improved compared to Res. However, the MIRes proposed in this paper achieves better results, and the increase in the amounts of parameters and computation is almost negligible. Compared with Res and IRes, the introduction of mixed convolution enables MIRes to have stronger multiscale feature extraction capabilities, so it can achieve better detection accuracy in multiscale ship target detection in ORSIs.

Table 6 shows the comparison results of the multiscale feature enhancement module and other feature enhancement modules. For fairness, RFB, EIRM [13], and the multiscale feature enhancement module are added to the same location on the basis of the improved backbone network. SFEM and MFEM in this paper act on the middle and low-level feature maps, respectively. Therefore, two RFBs and two EIRMs were added in the experiment to act on the middle and low-level feature maps. S-RFB represents adding RFB modules to the low-level feature map branch, and M-RFB represents adding RFB modules to the midlevel feature map. S-EIRM means adding EIRM to the low-level feature map branch, and M-EIRM means adding EIRM to the middle-level feature map. According to the results, it is obvious that, in the low-level feature map, the atrous convolution of the RFB with a large expansion rate may introduce a large amount of background, which will cause a decrease in accuracy. The scaling strategy of EIRM is also less accurate. SFEM only uses a combination of atrous convolution with an expansion rate of 1 and ordinary convolution, which enhances the feature description while suppressing the interference of background noise, and improves the accuracy of ship detection. For midlevel feature maps, MFEM also achieves better results than RFB and EIRM. Finally, the proposed multiscale feature enhancement module achieves higher accuracy than EIRM and RFB. Therefore, the strategy of using different enhancement modules for feature maps of different scales can achieve better results than the fixed feature enhancement strategy.

In order to verify the impact of the IOU loss function on the detection accuracy, this paper uses GIOU, DIOU, and CIOU to conduct comparative experiments. The experimental results are shown in Table 7. It is obvious that, in the algorithm of this paper, CIOU achieves the best effect compared to GIOU and DIOU. CIOU introduces the strategy of anchor box aspect ratio, which enables it to achieve higher accuracy than DIOU.

### 4.5. Ablation Experiments

To verify the effectiveness of each module, ablation experiments were implemented on the LEVIR-ship dataset.  Table 8 is the results of the ablation experiments. It is obvious that MIRes and the multiscale feature enhancement modules SFEM and MFEM proposed in this paper can effectively improve the detection accuracy of the baseline network YOLO v4. This proves that the improvements proposed in this paper can effectively improve the accuracy of multiscale ship detection in ORSIs. MIRes used improved mixed convolution and wider network structure, which greatly enhances the multiscale feature extraction capability of the backbone network. MFEM and SFEM act on the middle- and low-level feature maps to further enhance the feature description of ship targets, thereby improving the accuracy of ship detection. At the same time, SFEM, MFEM, and MIRes were added, and the method in this paper finally reached mAP of 79.55%. Compared with the baseline network, it has obtained a great improvement.

### 4.6. Extend Experiment

To further verify the effectiveness and scalability of our algorithm on other categories, this paper implements extended experiments on the NWPU VHR-10 dataset. The experimental results are shown in Table 9. AI, SH, ST, BD, TC, BC, GTF, HB, BR, and VH represent airplane, ship, storage tank, baseball diamond, tennis court, basketball court, ground track field, harbor, bridge, and vehicle, respectively. It can be seen from the results that the accuracy of the proposed algorithm for the overall mAP and ship category has reached the highest level. At the same time, it is extended to other categories, such as BD, TC, BC, GTF, HB, and BR. The algorithm in this paper is improved compared to YOLO v4.

Figure 16 is the comparison of the loss curve between the algorithm in this paper and the YOLO v4 algorithm on the NWPU VHR-10 dataset. Obviously, although the loss curve amplitude of the algorithm in this paper is large, the detection accuracy is steadily improved, while the loss value converges. The YOLO v4 algorithm converges faster and the curve is smooth, but its detection accuracy is low.

Figure 17 is the comparison of some detection results between the proposed algorithm and the YOLO v4 algorithm on the NWPU VHR-10 dataset. In order to reflect the scalability of the proposed algorithm in other categories, this paper selects images that contain different targets and are difficult to detect. The detection results contain a total of seven groups of images. Figures 17(a)–17(g) are the original images, Figures 17(h)–17(n) are the YOLO v4 detection results, and Figures 17(o)–17(u) are the detection results of the algorithm in this paper. Among them, some targets in Figures 17(a) and 17(b) are occluded by shadows, some targets in Figures 17(c) and 17(d) are not completely intercepted, and the colors of targets and backgrounds in Figures 17(e) and 17(f) are similar. Targets in Figure 17(g) are larger. According to the detection results of Figures 17(h)–17(n) and Figures 17(o)–17(u), it can be seen that YOLO v4 is prone to missed detection and false detection when detecting shadow-occluded targets, intercepted targets, and targets with similar background color and texture. The proposed algorithm can extract more multiscale feature information, and the multiscale feature enhancement module can further enhance the feature description and receptive field of the target and suppress the interference of background information. It has better detection results for multiscale targets in complex backgrounds.

## 5. Conclusion

To improve the accuracy of multiscale ship target detection in ORSIs, the multiscale feature enhancement ship target detection algorithm based on the one-stage algorithm YOLO v4 is proposed in this paper. Firstly, in order to improve the multiscale feature extraction capability of the backbone network, this paper improved the mixed convolution and proposed MIRes based on the improved mixed convolution. The MIRes are used to replace the Res in the deep CSP module. The wider network structure of the MIRes and the multikernel mixed convolution greatly enhance the feature extraction capability of the backbone network and the feature map receptive field. Secondly, the multiscale feature enhancement modules SFEM and MFEM are proposed, which act on the middle and low-level feature maps to enhance the feature map receptive field and feature information. Finally, comparative and extended experiments are implemented on the LEVIR-ship dataset and the NWPU VHR-10 dataset. The experimental results on the LEVIR-ship dataset show that the proposed algorithm achieves a 3.25% improvement compared to the baseline network and meets the requirements of implementation detection. At the same time, compared with the current relatively excellent feature enhancement modules, the multiscale feature enhancement module in this paper has achieved the best results. The experimental results on the NWPU VHR-10 dataset show that the proposed algorithm achieves a 3.56% improvement in the ship category compared to the baseline network. At the same time, it also achieved good results in the categories of base diamond, tennis court, basketball court, ground track field, harbor, and bridge.

## Figures and Tables

**Figure 1:** Display of ship target images in ORSIs. (a) Small-scale ship target. (b) Ship target obscured by clouds. (c) Ship targets against complex backgrounds.

**Figure 2:** Overall network structure diagram.

**Figure 3:** SPP module structure diagram.

**Figure 4:** CSP module structure diagram.

**Figure 5:** Comparison of (a) Res and (b) MIRes.

**Figure 6:** The proposed mixed convolutional structure diagram.

**Figure 7:** Example diagram of semantic information. The shallow feature maps are usually some corners and so on. The middle layer is part of the object. The deep layer is usually a whole object with rich semantic information.

**Figure 8:** SFEM structure diagram.

**Figure 9:** MFEM structure diagram.

**Figure 10:** Loss function limits. Green is the predicted box. Blue is the true box.

**Figure 11:** Schematic diagram of DIOU. *c* is the diagonal of the minimum bounding box of the real box and the predicted box, and *ρ* is the distance between the center points of the two.

**Figure 12:** Distribution of object locations and scales in the LEVIR-ship dataset. (a) Target location distribution. (b) Target scale distribution.

**Figure 13:** Distribution of object locations and scales in the NWPU VHR-10 dataset. (a) Target location distribution. (b) Target scale distribution.

**Figure 14:** Loss curve comparison chart. (a) YOLO v4 loss curve. (b) The loss curve of the algorithm in this paper.

**Figure 15:** Comparison of test results. The yellow arrow points to the targets of missed detection and false detection.

**Figure 16:** Comparison of loss curves. (a) YOLO v4 loss curve. (b) The proposed algorithm loss curve.

**Figure 17:** Comparison of detection results in the NWPU VHR-10 dataset. The yellow arrow points to the targets of missed detection and false detection.

**Algorithm 1:** Multiscale feature enhanced ship target detection.

**Algorithm 2:** K-means++ algorithm

**Table 1:** Res and MIRes network architecture and parameters.

	Res	MIRes
Input	13 × 13 × 512	13 × 13 × 512

Operation	$\left[\begin{array}{c} 1\times 1Conv\times 512\\ 3\times 3Conv\times 512 \end{array}\right]$	$\left[\begin{array}{c} 1\times 1Conv\times 3072\\ \left[\begin{array}{c} 1\times 1Dwise\times 1536\\ 3\times 3Dwise\times 768\\ \begin{array}{c} 5\times 5Dwise\times 384\\ 7\times 7Dwise\times 384 \end{array} \end{array}\right]\\ 1\times 1Conv\times 512 \end{array}\right]$

Output	13 × 13 × 512	13 × 13 × 512

13 × 13 × 512 represents the width, height, and number of channels of the feature map.

**Table 2:** The priori box size for the LEVIR-ship dataset and NWPU VHR-10 dataset.

Feature map	Receptive field	Detection object	Anchor box	
			LEVIR-ship	NWPU VHR-10
13 × 13	Large	Large	(77, 102), (104,138), (152,202)	(36, 27), (57,65), (130,121)
26 × 26	Medium	Medium	(31, 41), (45,60), (61, 81)	(22, 13), (16,21), (18, 39)
52 × 52	Small	Small	(8, 11), (13, 17), (21, 28)	(6, 8), (15, 8), (10, 16)

**Table 3:** the LEVIR-ship dataset with the experimental results.

Method	mAP (%)	FPS (s)
LARGE-RAM [38]	60.80	0.2
Faster RCNN [41]	79.0	6.4
EIRM-SGPANet [13]	77.82	51.7
YOLO v4	76.30	61.8
Ours	79.55	56.2

**Table 4:** Comparison of convolution kernel size and distribution method of mixed convolution.

Method	mAP (%)	Parameter (M)	BFLOPS (G)	FPS (s)
MIRes-3579	77.78	254	60.442	56.2
MIRes-1357	77.8	253	60.359	61.8
MIRes-3579exp	76.9	253	60.384	61.8
MIRes-1357exp (ours)	78.75	253	60.322	61.8

**Table 5:** Comparison of different residual blocks.

Method	mAP (%)	Parameter (M)	BFLOPS (G)	FPS (s)
Res (YOLO v4)	76.3	244	59.563	61.8
IRes	77.2	252	60.309	61.8
MIRes (ours)	78.75	253	60.322	61.8

**Table 6:** Comparison of feature enhancement modules.

Feature enhancement	mAP (%)	Parameter (M)	BFLOPS (G)	FPS (s)
S-RFB	77.73	254	61.873	56.2
S-EIRM	77.95	257	64.354	56.2
SFEM	79.21	247	64.791	61.8
M-RFB	78.26	257	61.872	56.2
M-EIRM	78.16	272	64.265	51.7
MFEM	78.55	267	65.55	56.2
S-RFB, M-RFB	76.52	258	63.423	56.2
S-EIRM, M-EIRM	76.79	276	68.297	51.7
SFEM, MFEM	79.55	271	70.778	56.2

**Table 7:** Comparison of loss functions.

Loss function	mAP (%)	FPS (s)
GIOU	77.69	56.2
DIOU	77.56	56.2
CIOU	79.55	56.2

**Table 8:** Ablation experiment.

MIRes	SFEM	MFEM	mAP (%)	Parameter (M)	BFLOPS (G)	FPS (s)
Baseline			76.3	244	59.563	61.8
√			78.75	253	60.322	61.8
	√		78.84	247	64.791	61.8
		√	77.18	258	64.791	56.2
√	√		79.21	256	65.55	61.8
√		√	78.55	267	65.55	56.2
	√	√	77.65	262	70.019	56.2
√	√	√	79.55	271	70.778	56.2

**Table 9:** Extended experimental results of NWPU VHR-10 dataset.

Method	AI (%)	SH (%)	ST (%)	BD (%)	TC (%)	BC (%)	GTF (%)	HB (%)	BR (%)	VH (%)	mAP (%)
FCOS [42]	90.47	73.72	90.36	98.94	89.38	80.82	96.74	87.91	61.92	88.16	85.84
SHDET [43]	100	81.36	90.90	98.66	90.84	82.57	98.68	91.11	76.43	89.82	90.04
FMSSD [44]	99.70	89.90	90.30	98.20	86.00	96.80	99.60	75.60	80.10	88.20	90.40
MRFF-RCA [40]	99.50	88.40	90.20	98.70	89.20	95.40	99.20	89.60	82.20	92.90	92.50
YOLO v4	99.97	87.16	98.54	97.38	97.73	94.54	99.65	82.67	77.61	93.42	92.87
Ours	99.93	90.72	98.45	97.67	99.66	96.45	99.80	83.55	83.64	91.69	94.17

## Data Availability

The research data come from the network public dataset. The NWPU VHR-10 dataset can be downloaded at https://www.heywhale.com/mw/dataset/5e9d2c33ebb37f002c618636. The LEVIR dataset can be downloaded at http://levir.buaa.edu.cn/Code.htm. The LEVIR-ship dataset and experiment results can be downloaded at https://pan.baidu.com/s/18n1KIsUOQiCGbPwDDPme6g?pwd=1111.
